The article "System Design and Simulation for Square Dance Movement Monitoring Based on Machine Learning" was published in 2022. Journal: Comput Intell Neurosci.

# System Design and Simulation for Square Dance Movement Monitoring Based on Machine Learning

**DOI:** 10.1155/2022/1994046

**Published:** 2022-05-19

**Authors:** Ping Lei

**Affiliations:** School of Physical Education, Chengdu Normal University, Chengdu 611130, Sichuan, China

## Abstract

Since the reform and opening, China's economy has grown rapidly, and people's living standards have improved significantly. As one of the most effective ways to implement national fitness, square dance has gradually become the main lifestyle of urban communities, an important part of China's sports construction, and an important indicator to reflect the fitness of the masses and the construction of a well-off society in an all-round way. On the other hand, with the rapid development of internet of things technology, many people can use intelligent bracelets based on machine learning technology to realize motion detection. This technology is also applicable in square dance, which is of great significance to exercise and protect health. This paper first reviews the research status of the internet of things communication protocol and cloud platform, then introduces and analyzes the MQTT communication protocol and Netty high-performance network framework, and studies the integration technology of the internet of things and machine learning. Then, according to the characteristics of the internet of things, a scheme to realize data preprocessing is proposed. The value to be completed is calculated based on the correlation of other attributes corresponding to the k-nearest neighbor model (KNN) and the regression model. Finally, the machine learning algorithm is used to train the results of the three models to obtain the final filling value. The whole scheme design allows the machine learning algorithm to obtain relatively high-quality data in the internal environment. This paper designs a sports monitoring data system for square dance by combining machine learning and internet of things technology, so as to promote national fitness.

## 1. Introduction

With the continuous growth of China's economy, the construction of urban civilization has been paid more and more attention by government departments at all levels. Since the reform and opening up, the pace of urban construction has accelerated, and urban communities have emerged rapidly, forming a unique urban culture [1]. Community residents use the vast and open space of the square to carry out various sports and cultural activities [2]. Due to its rich content, novel forms, and distinctive characteristics, square dance has gradually become the most popular fitness project [3]. It originates from social life and affects people themselves. It is a necessary form to promote the development of urban civilization. The development of square dance not only has a significant impact on urban civilization but also the basis of promoting the rapid growth of the urban economy [4]. With the aging development of square dance, some elderly people may be injured during exercise [5]. Therefore, this paper develops an intelligent bracelet based on machine learning and a data system, combined with the internet of things to monitor the exercise process [6]. Firstly, this paper uses basic research methods such as literature, questionnaire, and interview to investigate and analyze the physical status, exercise status, and physical and mental changes of community residents participating in the study [7]. In the square dance practice, the movement law and time period are studied and calculated [8]. In order to identify the action model, two classification algorithms with different complexity based on machine learning, SVM and deep neural network (established by one-dimensional CNN and LSTM, respectively), are proposed to adapt to different computing scenarios [9]. For cycle calculation, a method based on zero-crossing detection and wavelet transform is proposed to calculate the number of actions and the cycle of each action [10]. Then, a method that can fill the characteristic data system of the internet of things is proposed. The fill value is calculated through short-term correlation and other attribute correlation. Finally, the results of the three models are combined to form the final scheme to improve the filling accuracy. Finally, the more advantageous extreme machine learning (ELM) algorithm is selected as the research goal [11]. Based on de-elm, an online gp-elm is proposed, which increases the number of elm nodes hidden by jumping [12]. At the same time, it adopts the methods of dynamically determining the contribution of computing nodes with little negative impact and deleting relevant nodes according to the learning network structure, hoping to contribute to the movement monitoring process of square dance for the elderly, so as to promote comprehensive fitness [13].

## 2. Related Work

The literature provides an interface based on the LightGBM intelligent prediction module that can make the device have specific autonomous learning ability and provide an intelligent development idea for new internet of things devices [14]. The communication protocol is analyzed and studied in the literature [15]. Based on the specific needs, combined with artificial intelligence technology to solve the problems of cross-platform difficulty and fierce competition, an extremely reliable, high-performance, and scalable intelligent internet of things cloud platform is designed [16]. The platform can withstand massive concurrency, so as to realize cross-platform (high portability) operation, and can perform many functions such as predicting user behavior and intelligent device operation [17]. This paper proposes a design framework for encrypted verification MQTT message transmission, which can effectively improve the security of message transmission and then puts forward some suggestions based on the prediction and push module interface of the LightGBM algorithm [18]. The literature collected the relevant data in the general internet of things, simulated the designed scheme and algorithm with MATLAB software, and then compared some existing schemes. The experimental results show that compared with the traditional methods, the GP-ELM proposed in this paper has a certain accuracy while improving the training speed and can complete the task automatically [19]. Literature constructs the correlation between behavioral logic characteristics and interaction design elements. According to the different levels of correlation matching, the interactive design strategy of the old smart bracelet is proposed based on the four levels of functional content, information architecture, operation mode, and visual performance. According to the behavior characteristics of elderly users, the design strategy is changed into a specific interactive practice course, and then the interactive practice of designing an elderly intelligent bracelet is completed, and the possibility of methodology and strategy is verified by the usability test [20].

## 3. Theoretical Basis

### 3.1. Machine Learning

According to the similarity of algorithm functions, machine learning models can be divided into prediction, classification, grouping, neural network, deep learning, and other models.

Naive Bayes aims to calculate *P*(*a*|*b*), that is, the probability that event *a* will occur due to the probability that event *b* has occurred. In a classification model, *b* belongs to the sample of observation data, and *a* belongs to the category of prediction samples, that is, *P*(*a*|*b*) calculates the probability that *b* belongs to class *a*. The essence of naive Bayes is to use computational data, that is, according to our current data; constantly update the model parameters; and finally calculate the probability model of the category to which the training prediction sample belongs.

The expression of the naive Bayes formula is as follows:

(1) $$\begin{array}{c} P\left(C_{j}|D\right)=\frac{P\left(C_{j}\right)P\left(D|C_{j}\right)}{P\left(D\right)}, \end{array}$$

where *P*(*C*_*j*_ID): category *C* of document *D* to be classified; probability value *P*(DI*C*_*j*_): *C*, probability of document *D* appearing in the category; *P*(*C*_*j*_): probability of randomly selecting documents belonging to *C*_*j*_ category; and *P*(*D*): the probability of a document.

The expression of the linear regression model is

(2) $$\begin{array}{c} f\left(x_{i}\right)=\omega x_{i}+b, \end{array}$$

where *W* – weight matrix, *X*_*i*_ – sample point, and *B* – offset.

The *x* value can be input through the model to predict the *y* value. In order to make the prediction result more accurate, that is, make the difference between the predicted value *f*(*x*) and the known real value *y* as small as possible, so as to establish the cost function *J*(*w*), which is also called the loss function.

(3) $$\begin{array}{c} J\left(\omega ,b\right)=\underset{\omega ,b}{\min}{\sum \left(f\left(x_{i}\right)-y_{i}\right)}^{2}. \end{array}$$

The expression of the linear regression model is brought into the loss function to obtain

(4) $$\begin{array}{c} J\left(\omega ,b\right)=\underset{\omega ,b}{\min}\sum^{}{\left(y_{i}-\omega x_{i}-b\right)}^{2}. \end{array}$$

The least-square method is used to optimize the cost function, and through continuous iteration, a curve that best fits the training data is found. Assuming that the function is optimal and the cost function is 0, find the partial derivative and solve the equations:

(5) $$\begin{array}{c} \frac{\partial J\left(\omega ,b\right)}{\partial \omega }=2\overset{m}{\underset{i=1}{\sum }}\left(\omega x_{i}^{2}-x_{i}\left(y_{i}-b\right)\right),\\ \frac{\partial J\left(\omega ,b\right)}{\partial b}=2\overset{m}{\underset{i=1}{\sum }}\left(b-\left(y_{i}-\omega x_{i}\right)\right)=2\left(mb-\overset{m}{\underset{i=1}{\sum }}\left(mb-\overset{m}{\underset{i=1}{\sum }}\left(y_{i}-\omega x_{i}\right)\right)\right). \end{array}$$

Since the extreme value of the function is obtained when the partial derivative is 0, make the above formula equal to 0, and solve the equations to obtain

(6) $$\begin{array}{c} b=\bar{y}-\omega \bar{x}=\frac{1}{m}\overset{m}{\underset{i=1}{\sum }}y_{i}-\omega \frac{1}{m}\overset{m}{\underset{i=1}{\sum }}x_{i},\\ \omega =\frac{\sum_{i=1}^{m}y_{i}\left(x_{i}-\bar{x}\right)}{\sum_{i=1}^{m}x_{i}^{2}-{\bar{x}}^{2}}=\frac{\sum_{i=1}^{m}y_{i}\left(x_{i}-1/m\sum_{i=1}^{m}x_{i}\right)}{\sum_{i=1}^{m}x_{i}^{2}-{\left(1/m\sum_{i=1}^{m}x_{i}\right)}^{2}}, \end{array}$$

where $\bar{x}$is the mean value of sample point *x* and $\bar{y}$ is the mean value of sample point *y*.

From this, we get the optimal parameter *W* of the linear regression model and bring it into the initial formula to get the expression of the model. In addition, in order to make the model have better overall performance, that is, the model has specific fault tolerance, regular items must be added to the model.

### 3.2. Internet of Things Communication Protocol

The communication protocol is the communication code established by both sides of communication, and it is also a rule that must be observed. In the communication of the internet of things; the communication protocol is often based on TCP/IP protocol, which is responsible for the data exchange between devices. The widely used communication protocols are REST/HTTP, XMPP, COAP, and MQTT.

1. REST/HTTP encapsulates the Internet Service API, simplifies the architecture of the Internet system, and realizes the low-latency and poor coupling data interaction between the client and the server through the open REST API.
2. XMPP is an XML-based protocol with strong scalability, flexibility, high integration, and ease of use. XMPP-based applications can use existing resources to expand subscription and publishing functions, and developers can easily add additional functions to the configured XMPP system.
3. CoAP is an application layer protocol, short for constrained application protocol. It can be used in6LoWPAN protocol stack and communication networks with limited resources.
4. MQTT is a communication protocol developed by IBM for telemetry message transmission queue. It is the abbreviation of message queuing telemetry transport. Its dissemination mode adopts publishing and subscription. MQTT is suitable for low bandwidth and insecure networks. This network architecture requires a message proxy server, so it is not suitable for communication between devices.

The characteristics of existing IoT communication protocols are compared as shown in Table 1.

By introducing the above protocols and analyzing the four communication protocols in Table 1, MQTT and COAP are compared with REST/HTTP and XMPP protocols in terms of generality, compatibility, scalability, security, and bandwidth use. It is concluded that the real-time performance of MQTT is better than COAP.

The data packet of the MQTT protocol is divided into three parts: fixed header, variable header, and payload. The structure of the MQTT package is shown in Table 2:

MQTT is divided into 14 different messages according to functions, as shown in Table 3.

## 4. Optimization Design of Internet of Things Data System Based on Machine Learning

### 4.1. Internet of Things Data Preprocessing

Traditional methods usually use hand-made features to model the time-series prediction problem and use well-designed regressors to predict. A recurrent neural network (NNR) is selected because it can model long-term historical information over time. Although several standard LSTM variants have been proposed recently to achieve long-term dependence, large-scale analysis shows that none of them can improve the processing performance for this problem. Therefore, we solve the problem of long-term dependence by replacing simple RNN units with LSTM neural structures in a cyclic neural network. LSTM is a special type of RNN. Through its closed structure, including forgetting gate, input gate, and output gate, LSTM can remember what should be remembered and forget what should be forgotten. In particular, “forgetting gate” is the first LSTM operator that decides to use the sigmoid function to delete the last time-step information, and it is also the key operator of the gate structure. First, we define attention to weight as

(7) $$\begin{array}{c} W=\left(W^{1},W^{2},\ldots ,W^{L}\right). \end{array}$$

Through these focus weights, we can sample the input data based on importance:

(8) $$\begin{array}{c} \tilde{X_{t}}=\left(x_{t}^{1}W^{1},x_{t}^{2}W^{2},\ldots ,x_{t}^{L}W^{L}\right). \end{array}$$

In addition, we can understand the nonlinear mapping function of the calculation process in the LSTMS unit through the following formula:

(9) $$\begin{array}{c} i^{t}=\sigma \left(W_{xi}\tilde{X_{t}}+W_{hi}h^{t-1}+W_{ci}c^{t-1}+b_{i}\right),\\ f^{t}=\sigma \left(W_{xf}\tilde{X_{t}}+W_{hf}h^{t-1}+W_{cf}c^{t-1}+b_{f}\right),\\ c^{t}=f^{t}c^{t-1}+i^{t}\tanh\left(W_{xc}h^{t-1}+W_{hc}c^{t-1}+b_{c}\right),\\ o^{t}=\sigma \left(W_{xo}\tilde{X_{t}}+W_{ho}h^{t-1}+W_{co}c^{t-1}+b_{o}\right),\\ h^{t}=o^{t}\tanh\left(c^{t}\right), \end{array}$$

where ( ) refers to the activation function of *S*-type and *W*-matrix, in which the connection weight between two units is double subscript. It indicates the input gate state of the current time step, *f*^*t*^ is the state of the forgotten gate, *c*^*t*^ is the cell, *t*^*t*^ is the output gate state, and *h*^*t*^ is the output hidden layer state of the current time step. Finally, we can take the last element of the output vector *h*^*t* − 1^ as the predicted value. It can be expressed as follows:

(10) $$\begin{array}{c} {\tilde{y}}^{t}=h^{t-1}. \end{array}$$

The final output value can be associated with the vector as follows:

(11) $$\begin{array}{c} \tilde{yT}=\left({\tilde{y}}^{1},{\tilde{y}}^{2},\ldots ,{\tilde{y}}^{T}\right). \end{array}$$

### 4.2. Optimization Method of Limit Learning Machine

Compared with the original algorithm, the start-up phase has not changed. The optimization aspects of this paper are as follows: first, when adding nodes, set a large number so that each temporary increase of nodes has more values. Second, a simple method to calculate the contribution is added in the process of node removal, and according to these contributions, two methods are used to accurately eliminate the parts that are almost inefficient. The last is the internet of things data adaptation. The continuous characteristic of the online limit learning machine is based on the online limit learning machine, and the steps are added so that the elm parameters can be updated with the data flow. The specific steps are as follows: Parameters of randomly generated hidden nodes (*a*_1_, *b*_1_) ∈ *R*^*d*^ × *R*.

Calculate the output matrix of the hidden layer as follows:

(12) $$\begin{array}{c} H=\left[\begin{array}{c} G\left(a_{1},b_{1},x_{1}\right)\\ \vdots \\ G\left(a_{1},b_{1},x_{N}\right) \end{array}\right]. \end{array}$$

Calculate the optimal output weight as follows:

(13) $$\begin{array}{c} \beta =H^{†}T, \end{array}$$

where *H*^†^ is the generalized inverse of *H* and *t* is the objective matrix. So we get the initial function Ψ1 and related error *E*_1_ as follows:

(14) $$\begin{array}{c} \Psi_{1}\left(x\right)=\beta_{1}G_{1}\left(x\right),E_{1}=\Psi_{1}-t. \end{array}$$

Hide nodes rise and delete (maximum hidden node number Lmax, demand error rate *ε*).

Generate *m* hidden node parameters and add them to the current model, and then according to the iterative formula

(15) $$\begin{array}{c} \beta_{k+1}=H_{k+1}^{†}T=\left[\begin{array}{c} U_{k}\\ D_{k} \end{array}\right]T,\\ D_{k}={\left(\left(I-H_{k}H_{k}^{†}\right)\sigma H_{k}\right)}^{†},\\ U_{k}=H_{k}^{†}-H_{k}^{†}\sigma H_{k}D_{k}. \end{array}$$

Set *r* = 0, where *k* is the index representing the number of data blocks presented to the network. Give the (*r* + 1) new observation:

(16) $$\begin{array}{c} S_{r+1}=\left\{\left(\begin{array}{c} x_{i},t_{i} \end{array}\right)|x_{i}\in R^{n},t_{i}\in R^{m},i=\left(\overset{r}{\underset{j=0}{\sum }}n_{j}\right)+1\cdots \overset{r+1}{\underset{j=0}{\sum }}n_{j}\right\}, \end{array}$$

where *n* represents the number of newly obtained observations in the *r* block.

Calculate the output matrix *h*_*r* + 1_ of some hidden layers as follows:

(17) $$\begin{array}{c} h_{r+1}=\left[\begin{array}{ccccccc} G\left(a_{1},\right. & b_{1}, & \left.x_{N_{r+1}}\right) & \cdots & G\left(a_{\tilde{N}},\right. & b_{\tilde{N}}, & \left.x_{N_{r+1}}\right)\\ \; & \vdots & \; & \ddots & \; & \vdots & \;\\ G\left(a_{1},\right. & b_{1}, & \left.x_{N_{r+1}}\right) & \cdots & G\left(a_{\tilde{N}},\right. & b_{\tilde{N}}, & \left(x_{N_{r+1}}\right) \end{array}\right]. \end{array}$$

Calculate the output weight matrix *β*_*k* + 1_ as follows:

(18) $$\begin{array}{c} \left\{\begin{array}{c} {\hat{\beta }}^{\left(r+1\right)}={\hat{\beta }}^{\left(r\right)}+P_{r+1}h_{r+1}^{⊤}\left(t_{r+1}-h_{k+1}{\hat{\beta }}^{\left(r\right)}\right),\\ P_{r+1}^{-1}=p_{r}^{-1}+h_{r+1}^{⊤}h_{r+1}, \end{array}\right) \end{array}$$

where *P*_*r*_ is the update matrix.

### 4.3. Analysis of Optimization Effect of Internet of Things Data System

The proposed GP-ELM algorithm is compared with the original elm and different derived versions of OS-ELM, EI-ELM, D-ELM, and EM-ELM. The specific process of the experiment is as follows.

The proposed algorithm is compared with the original elm algorithm, and the results are shown in Figure 1.

As can be seen from Figure 1, the algorithm proposed in this paper first completes the task of automatically generating the number of hidden nodes, which is not conducive to increasing the training time and has a significant improvement in accuracy. This is because the algorithm proposed in this paper removes some unimportant hidden nodes that have little impact on the results after adding nodes each time, so the remaining nodes are more important nodes, which have a great impact. Therefore, the algorithm proposed in this paper obtains high accuracy when the nodes are relatively small.

Before the algorithm proposed in this paper, several algorithms try to solve similar problems, so they are compared with this algorithm, as shown in Figure 2.

We have chosen several algorithms used in practical applications: logical regression, SVM, and random forests, and in the same environment, the proposed algorithm is transversely comparable, as shown in Figure 3.

The data obtained from the experiment can compare the training accuracy: the algorithm proposed in this article is very close to the two classifiers SVM and random forests, accurate rates are much higher than the general logic regression classifier, which shows that the algorithm has certain reliability. Training time comparison: Two strong classifications have selected the training method of multicycle training parameters to achieve the final accuracy, making the training time be long. Logic regression uses a gradient reduction method and a long-term training method. The algorithm proposed in this paper uses the least squares to obtain the optimal solution. The required full matrix calculation and total calculation amount are relatively small, so the proposed algorithm has the advantage of training time. About parameter settings: SVM takes a long time to use cross-validation to select the optimal parameters; the random forest is a very good overall algorithm and do not need to do too many parameter debugging; the control variable is easier to choose; logic regression can only learn only control and debugging; and the algorithm proposed herein will adjust the control parameters to the network to achieve the effect of the control parameter automatically generated by continuously adding nodes to the network.

## 5. Square Dance Monitoring Method Based on Related Technology

### 5.1. Analysis of the Status Quo of Square Dance Exercise

#### 5.1.1. Research Method

*(1) Document Information Method*. Through a variety of methods, we fully grasp the various relevant literature materials for current urban community sports and square dance research. The main way is to take community sports and square dance as keywords, search about 121 documents online in the full-text database of Chinese journals, and select more than 40 papers to provide theoretical basis for the design, conception, and analysis of papers.

*(2) Questionnaire Survey*. Through reading a large number of literature that refer to a large number of community sports research materials, this paper combines the characteristics of research purposes and square dance, the initial table of the “questionnaire” in the test area, and urban community square dance participants. The prepared questionnaire content is finally determined after the authority review.

In order to ensure the effectiveness of the questionnaire, we distribute them to eight aerobics and gymnastics experts from the test area sports college, including five professors and associate professors. The results of the valid survey are shown in Table 4.

The distribution and retrieval of the questionnaire: the questionnaire random survey is conducted by participants from 16 communities from the test area square dance. 1,000 questionnaires were issued and 952 were recovered. The survey recovery is 95.20%, with 916 effective questionnaires, and the actual effective questionnaire is 96.22% (see Figure 4 for details).

#### 5.1.2. Research Results

The gender, age, educational level, and occupation of the participants in the national square dance in the study area were investigated. The basic information of the survey is as follows: from the perspective of gender, there are great differences in the proportion of men and women in the community participating in the national square dance in the test area. In terms of age, the participants aged 46–60 are the most, up to 41.03%, indicating that the elderly and middle-aged are the main groups participating in exercise (see Table 5 for details).

The survey found that the main motivation for participating in the community square dance in the test area was fitness, accounting for 68.99%, followed by entertainment and leisure, fitness and weight loss, and medical care, accounting for 47.27%, 30.46%, and 20.63%, respectively, followed by social interaction, pursuit of fashion, and others, accounting for 9.17%, 5.79%, and 0.87%, respectively, as shown in Figure 5.

Sports help promote the physical and mental development of athletes. According to the survey, the physical and mental changes brought by the national square dance to the participants in the test area are as follows. The first three are as follows: improving physical fitness and enriching life, improving sleep, preventing diseases and alleviating fatigue, accounting for 46.41%, 34.85%, and 23.70%, respectively. Through square dance exercises, the physical and mental health of participants has been well promoted and developed, which is an important driving force for them to continue to participate in exercise (see Table 6 for details).

### 5.2. System Design

The hardware components of the experimental system developed herein include bracelets, wireless access points (APs), and PCs, as shown in Figure 6. The main hardware components are data acquisition nodes, which can wear bracelets, including lithium battery power modules and downlink components, STM32F051K86 microcontrollers, ESP8266 communication modules, and MPU9250 behaviors based on MEMS inertia components. The bracelet plays a role in collecting and filtering motion data, calculating, and transmitting data to the host computer. Furthermore, the hardware also includes an AP and a PC for data processing: the AP is responsible for data communication between the bracelet and the PC, and the PC is responsible for running the receiving algorithm and processing data.

In multiuser motion monitoring systems, motion monitoring system software is used to perform data communication, motion start detection, data preoperation, pattern identification, cycle calculation, and visualization. The action identification algorithm and cyclic calculation algorithm involved herein are implemented in software. The relationship between different software components is shown in Figure 7. First, data transmission, automatic detection start, and stop action are performed. Next, the data pretreatment or feature extraction is performed, and the action model is identified. Finally, the number of cycles and frequency calculations are calculated using the correlation algorithm. After the above process is completed, the experimental results are shown in an image form.

### 5.3. Action Monitoring and Handling Methods

#### 5.3.1. Data Preprocessing

Different from the traditional machine learning algorithms that need feature extraction or feature selection, the deep learning network can extract high-level data segments by combining lower-level features, which has a stronger understanding ability, so it does not need to extract features manually. However, this does not mean that the data used for deep learning do not need any processing. As mentioned above, the original data generated by the behavior sensor used in this paper has nine axes, and each axis has a time series. For most deep learning structures, time series processing only accepts one-dimensional signals, so the original nine time series are not directly sent to the deep learning network for processing. Therefore, the original data must be preprocessed in order to convert it from nine-axis data to single-axis data.

The method used in this paper is to connect the data to nine axes in turn. The behavior module collects nine values every sampling hour, that is, the speed, angular velocity, and Euler angle of *X*-, *Y*-, and *Z*-axis, so that the length of the nine axes of the final data is the same, that is, at the same sampling point. After connecting the endpoints from beginning to end, the total length of the data will be nine times the original length. In this process, no information is lost, but the data conversion from nine axes to one axis meets the requirements of the deep learning framework.

#### 5.3.2. Action Counting and Cycle Calculation Method

When selecting the sensitive axis, this paper first excludes three angular axes (Euler angles) and only selects one of the other six axes as the sensitive axis for inspection. There are two reasons: first, for the original signal, waveform changes usually occur in some of the nine axes, which are concentrated on the three angular axes. For example, suppose the angle of an axis increases from 0. If it rises to +180° and continues to increase, the angle will suddenly change to −180°. This phenomenon is caused by the angle calculation method of the behavior module itself, which is unfavorable to the calculation of the time period. Therefore, the interference of three angles should not be included in the selection of sensitive axis. The following is the specific method of selecting a sensitive axis:

(19) $$\begin{array}{c} A={\left[A_{1},A_{2},\cdots ,A_{6}\right]}^{T},\\ S_{i}^{2}=\frac{1}{m}\left[{\left(A_{11}-{\bar{A}}_{i}\right)}^{2}+{\left(A_{i2}-{\bar{A}}_{i}\right)}^{2}+\cdots +{\left(A_{im}-{\bar{A}}_{i}\right)}^{2}\right],\\ i^{\prime }=\underset{i}{\arg\max}S_{1}^{2}, \end{array}$$

where *a* is the vector representation of the original data on the *I*-axis and *M* is the number of data sampling points, that is, the length of the data. This method calculates the difference between each axis. The serial number of the axis with the largest difference is *I*, so the *I*-axis is the selected sensitive axis. Through the sensitive axis selection, calculation, and time calculation methods, it only needs to calculate on one axis, which not only improves the calculation efficiency but also achieves higher accuracy.

Combined with the characteristics of zero-crossing detection and wavelet transform, a method to calculate action and time is proposed. This method eliminates the interference caused by limb trembling or other noise and can effectively count the number of reciprocating movements of limbs. The process is as follows:

(20) $$\begin{array}{c} C_{\psi }=\underset{R}{\int }\frac{{\left|\hat{\psi }\left(\omega \right)\right|}^{2}}{\left|\omega \right|}d\omega \;<\infty . \end{array}$$

Ψ(*t*) is called a wavelet base. The wavelet base used in this paper is cgau wavelet, which is a complex form of a Gauss wavelet. When wavelet base Ψ (t) is scaled or translated, we can get the wavelet sequence, namely:

(21) $$\begin{array}{c} \psi_{\left(a,b\right)}\left(t\right)=\frac{1}{\sqrt{\left|a\right|}}\psi \left(\frac{t-b}{a}\right),a,b\in R;a\neq 0, \end{array}$$

where *a* is the scale factor of wavelet transform and *b* is the translation factor.

For the selected key axis signal *f*(*t*) ∈ *L*^2^(*R*), the continuous wavelet transform is

(22) $$\begin{array}{c} W_{f}\left(a,b\right)=\langle f,\psi_{a,b}\rangle ={\left|a\right|}^{-1/2}\underset{R}{\int }f\left(t\right)\psi \left(\frac{t-b}{a}\right)dt\;. \end{array}$$

Inverse transform to

(23) $$\begin{array}{c} f\left(t\right)=\frac{1}{C_{\psi }}\overset{\infty }{\underset{-\infty }{\int }}\overset{\infty }{\underset{-\infty }{\int }}\frac{1}{a^{2}}W_{f}\left(a,b\right)\psi \left(\frac{t-b}{a}\right)da\;db. \end{array}$$

After the wavelet transform of the key axis signal, the wavelet coefficient matrix *A*_*m* × *n*_ is obtained, where *n* represents the number of layers of wavelet transform and *M* represents the number of sampling points, that is, the signal length.

For each,

(24) $$\begin{array}{c} a_{ij}\in A_{m\times n},0<i\leq m,0<j\leq n,i\in N,j\in N. \end{array}$$

Wavelet energy matrix *P* is

(25) $$\begin{array}{c} P=\left[\begin{array}{cccc} a_{11}{\;}^{2} & a_{12}{\;}^{2} & \ldots & a_{1n}{\;}^{2}\\ a_{21}{\;}^{2} & a_{22}{\;}^{2} & \ldots & a_{2n}{\;}^{2}\\ \vdots & \vdots & \ddots & \vdots \\ a_{m1}{\;}^{2} & a_{m2}{\;}^{2} & \ldots & a_{mn}{\;}^{2} \end{array}\right], \end{array}$$

where *N* represents an integer (the same below) and the energy matrix *Р*. The elements represents the amplitude of each harmonic component.

Next, use the vector as follows:

(26) $$\begin{array}{c} C=\left\{c_{1},\cdots ,c_{m}|c_{l}=\underset{k}{\arg\max}\left(p_{lk}\right)\right\}1\leq l\leq m,1\leq k\leq n;l,k\in N. \end{array}$$

That is the position where the component with the largest harmonic intensity appears at each time, that is, the position wavelet scale of the standard frequency of the sensor signal. *p*_*l*_ represents the *l*-th row of matrix *P*, and *p*_*lk*_ represents the element *K* of row *P*.

### 5.4. Analysis of Research Results

#### 5.4.1. Test Effect Analysis

In this system, the data transmission between the basic data forwarding station and Alibaba cloud server is based on HTTP protocol, which ensures the stability of data transmission. Therefore, the reliability of the system depends on the packet loss rate of wireless transmission between the data acquisition terminal and the database station. The packet loss rate is an important index to evaluate the quality of data links in wireless sensor networks, especially affected by factors such as distance and transmission time. The following are tests at different distances and times.

1. Test conditions: the wireless transmission power is adjusted to the maximum, and the transmission rate is 2 kbps.
2. Test method: when packet loss retransmission is turned on and off, the specific conditions of transmission distances of 500 meters, 1,000 meters, and 1,500 meters are tested on sunny, cloudy, and rainy days, respectively. The test results are shown in Figure 8.

Next, the experiment takes the dumbbell bending action as an example, repeats it 50 times, calculates the times and cycles according to the sensitive data on its axis, and finally compares the measured value with the actual value and checks it. The calculated and real values of 50 actions in this experiment are shown in Figure 9. The dotted line marked with a square is the measured value obtained by the cyclic calculation method; the solid line marked with a triangle is the real value recorded on the timer; the vertical axis is the action cycle in seconds; and the horizontal axis is the action times.

Firstly, from the length of the two numerical curves, it can be seen that the algorithm is very accurate, and the statistical results of 50 times are completely consistent with the real value. Secondly, the two numerical curves fit well as a whole, with an average error of only 0.08 s and an average error rate of 4.03%. The maximum error of the calculation result is 0.25 s; the maximum error rate is 13.5%; and it only appears at the end of the curve. Therefore, experiments show that the overall effect of zero-crossing detection and wavelet analysis method is good. When the number of actions is large, action counting and cycle calculation can be more accurate.

#### 5.4.2. User Satisfaction Analysis

Six elderly users were selected for the use test, and the running time of the tester to complete the task was recorded. The statistical results are shown in Table 7.

This assessment is mainly carried out from the four aspects of the visual performance, operation mode, task process, and function content of the smart bracelet. The five-level scale of the Likert scale is evaluated and counted, and the score is −2, −1, 0, 1, 2, which is very dissatisfied, unsatisfactory, satisfactory, satisfactory, and very satisfied, respectively.  Table 8 shows the satisfaction score statistics of the older user.

## 6. Conclusion

The development of the square dance in the research area is in line with the big trend of China's national fitness, which is conducive to the implementation of the Chinese national fitness program, which is also in line with the status quo of community sports in the research area, which not only reflects many advantages but also extensive market demand, but people's sports health is not guaranteed, so this paper has developed a smart bracelet based on machine learning and internet of things technology to obtain the basic state of the research area square dance. Through research analysis, then combined with the Internet, machine learning, and artificial technology, the design scheme is determined to provide the LightGBM intelligent predictive module interface based on the cloud platform so that the MQTT message middleware can call the interface and respond to the prediction result so that the device has specific autonomous learning capabilities, then select the machine ultimate learning machine ELM learning algorithm, and propose an online GP-ELM based on DE-ELM. ELM increases the use of computing nodes to eliminate almost no effect on the value of the calculation node, which improves the processing speed of the smart bracelet and hopes to help the square dance.

## Figures and Tables

**Figure 1:** Comparison of GP-ELM with ELM and OS-ELM.

**Figure 2:** Comparison of GP-ELM and EI-ELM, D-ELM, and EM-ELM.

**Figure 3:** Comparison with existing algorithms.

**Figure 4:** General situation of questionnaire distribution of national square dance participants in the test area.

**Figure 5:** Motivation of participants of national square dance in the community in the test area (multiple choice; *N* = 916).

**Figure 6:** Experimental system hardware composition.

**Figure 7:** Software structure box.

**Figure 8:** Packet loss rate test.

**Figure 9:** Action count and cycle calculation results.

**Table 1:** Comparison of internet of things communication protocols.

---	CoAP	XMPP	REST/HTTP	MQTT
Abstract	Request/reply	None	Request/reply	Pub/sub
QOS	Confirm or nonconfirmation message	None	Guarantee by TCP	3
Performance	100 req/S	No test data	100 req/s	1,000 msg/sub
Transport layer	UDP	TCP	TCP	TCP
Subscribe control	Support multicast address	None	None	Holiday matching topic subscription
Coding	Binary	XML text	Ordinary text	Binary
Safety	None	TSL data encryption	SSL and TLS	Username password, SSL data encryption

**Table 2:** MQTT packet composition.

Fixed header	It must exist and describe packet information. And the content needs to include the type of message and the level of the message.
Variable header	It is necessary to determine if it exists based on the fixed header message type.
Payload part	Where the communication data is stored, the content is included.

**Table 3:** MQTT message type.

Name	Value	Flow	Description
CONNECT	1	Client to the server	Client request connection server
CONNACK	2	Server to the client	Server confirming connection request
PUBLISH	3	Client and server two-way	Making an announcement
PUBACK	4	Server to the client	QoSL release confirmation
PUBREC	5	Server to the client	Qos2 release
PUBREL	6	Server to the client	QoS2 release
PUBCOMP	7	Server to the client	QoS2 release completion
SUBSCRIBE	8	Client to the server	Client subscription message
SUBACK	9	Server to the client	Confirm subscription
UNSUBSCRIBE	10	Client to the server	Cancel subscription request
UNSUBACK	11	Server to the client	Cancel subscription confirmation
PINGREQ	12	Client to the server	Ping request
PINGRESP	13	Client to the server	Ping reply
DISCONNECT	14	Client to the server	Clients disconnected

**Table 4:** Validity survey on the questionnaire (*N* = 8).

Overall evaluation	Very suitable	Suitable	Substantial	Unwell	Very uncomfortable
Number of people	0	1	7	0	0
Proportion (%)	0	12.5	87.5	0	0

**Table 5:** Gender and age distribution of participants in the national square dance in the community in the test area (*n* = 916).

---	Gender		Age				
	Male	Female	<15	16–30	31–45	46–60	>61
Number of people	199	717	33	115	242	375	152
Proportion (%)	21.63	78.37	3.48	12.44	26.32	41.03	16.73

**Table 6:** Physical and mental changes of participants in the national square dance in the community in the test area (multiple choices; *N* = 916).

Physical and mental change	Number	Proportion (%)	Sorting
Improve physical physique and make life more fulfilling	420	46.41	1
Create pleasant physical and mental conditions and relieve disease	177	19.74	4
Enhance appetite and promote memory	144	15.77	6
Improve sleep and reduce pressure	315	34.85	2
Tao Ye, improve the body	154	16.87	5
Prevent and treat diseases and relieve fatigue	216	23.70	3
Improve confidence and broaden people	108	11.80	7
Others	20	2.31	8

**Table 7:** Statistics of availability test time (s).

Tester	Design practice interface prototype			Existing smart bracelet interface		
	Task 1	Task 2	Task 3	Task 1	Task 2	Task 3
Test 1	46	16	38	56	28	55
Test 2	38	27	43	62	33	53
Test 3	42	27	32	47	22	47
Test 4	53	16	57	68	37	62
Test 5	47	28	56	75	46	41
Test 6	35	21	44	55	27	78
Time up limit	53	28	59	75	48	78
Time down limit	37	16	32	56	23	41
Average time	42.7	22.6	45.1	60.6	32.6	56.1

**Table 8:** Satisfaction score statistics.

First-class indicator	Secondary indicators	Test 1	Test 2	Test 3	Test 4	Test 5	Test 6	Mean
Visual performance	Style	1.0	1.0	2.0	0	1.0	2.0	1.15
	Color	1.0	2.0	0	1.0	1.0	2.0	1.15
	Text recognition	1.0	2.0	2.0	0	0	1.0	1.00
	Icon recognition	2.0	1.0	1.0	1.0	2.0	1.0	1.31

Operation method	Convenient operation	1.0	2.0	2.0	2.0	2.0	2.0	1.48
	Comfort	2.0	2.0	2.0	1.0	1.0	2.0	1.65
	Smooth operation	2.0	1.0	0	2.0	0	2.0	1.15

Task process	Slow process	2.0	1.0	1.0	−1.0	0	2.0	0.82
	Definitely	2.0	1.0	2.0	2.0	2.0	1.0	1.65
	Easy to learn	0	0	2.0	2.0	1.0	2.0	1.15
	Easy memory	−1.0	2.0	1.0	2.0	2.0	0	1.00

Functional content	Meet demand	2.0	1.0	1.0	0	2	1.0	1.15
	Attractive	1.0	2.0	−2.0	2.0	2.0	1.0	1.00

## Data Availability

The data used to support the findings of this study are available from the corresponding author upon request.
